The article "High-Calcium Microenvironment during the Development of Kidney Calculi Can Promote Phenotypic Transformation of NRK-52E Cells by Inhibiting the Expression of Stromal Interaction Molecule-1" was published in 2022. Journal: Biomed Res Int.

# High-Calcium Microenvironment during the Development of Kidney Calculi Can Promote Phenotypic Transformation of NRK-52E Cells by Inhibiting the Expression of Stromal Interaction Molecule-1

**DOI:** 10.1155/2022/2350198

**Published:** 2022-03-01

**Authors:** Li-Sha Li, Yun-Peng Zhu, Qi-Dong Xia, Shao-Gang Wang, Deng He

**Affiliations:** ^1^Department of Urology, Tongji Hospital, Tongji Medical College, Huazhong University of Science and Technology, No. 1095 Jiefang Avenue, Wuhan, 430030 Hubei, China; ^2^Department of Thoracic Surgery, Tongji Hospital, Tongji Medical College, Huazhong University of Science and Technology, No. 1095 Jiefang Avenue, Wuhan, 430030 Hubei, China; ^3^Department of Gynecology and Obstetrics, Tongji Hospital, Tongji Medical College, Huazhong University of Science and Technology, No. 1095 Jiefang Avenue, Wuhan, 430030 Hubei, China

## Abstract

**Objective:**

To explore whether Stromal Interaction Molecule-1 (STIM1) participates in the phenotypic transformation of NRK-52E cells under high-calcium microenvironment.

**Materials and Methods:**

NRK-52E cells were treated with high concentration of calcium. The viability and apoptosis of cells were detected by CCK-8 (cell counting kit-8) and flow cytometry, respectively. The expression changes of phenotypic marker proteins (E-cadherin and OPN) and calcium channel proteins (STIMl and Orai1) in high-calcium environment were detected by western blotting and real-time quantitative polymerase chain reaction. The expression of STIMl protein in NRK-52E cells was upregulated and downregulated by plasmid-STIM1 and plasmid-shRNA-STIMl, respectively. The expressions of phenotypic marker proteins after upregulation or downregulation of STIMl were detected again. Besides, the intracellular calcium concentrations of NRK-52E cells in different treatments were detected by flow cytometry.

**Results:**

High-calcium microenvironment can promote the phenotypic transformation and the adhesion of calcium salts in NRK-52E cells and simultaneously suppress the expression of STIMl protein in NRK-52E cells. Downregulation of STIMl protein could also promote the phenotype transformation, while both the gene silence of matrix gla protein (MGP) and overexpression of STIMl showed reverse results.

**Conclusion:**

STIMl protein plays an important role in promoting phenotypic transformation of NRK-52E cells in high-calcium microenvironment.

## 1. Introduction

Kidney stone, as one of the most common diseases in urology, seriously endangers public health [1, 2]. In China, approximately one in 17 adults suffers from kidney calculi [3]. Due to environmental pollution, eating habits, and so on, the incidence rate has been rising year by year [4]. In addition, the high rate of recurrence also significantly increases the physical and psychological stress of patients with calculi [5]. According to epidemiological reports, nearly two-thirds of newly diagnosed patients with calculi will recur in their lifetime [5, 6].

The occurrence of kidney calculi is closely related to the high-calcium microenvironment in renal papilla [7]. According to Randall's calcium plaque theory, Randall's calcium plaque is the key site of calculi formation and anchoring, and its essence is calcification originating from renal papillary interstitium [8, 9]. Some researchers believe that renal papillary interstitial calcification is caused by the phenotypic transformation of renal tubular epithelial cells. Epithelial cells in renal papilla differentiate into osteoblasts under high calcium, hypoxia, and other microenvironments [10]. After phenotypic transformation, the ability of cells to adhere to crystals is significantly increased, which becomes the starting point of renal papillary calcification and eventually leads to the formation of the Randall calcium plaque. However, the mechanism of phenotype transformation of epithelial cells induced by high-calcium microenvironment is still lack of relevant research.

STIM1 is a single transmembrane protein located on endoplasmic reticulum, and its N-terminal is in the lumen of endoplasmic reticulum, which can sense the change of intracellular calcium concentration through endoplasmic reticulum [11]. Furthermore, STIM1 can regulate the intracellular calcium concentration through CRAC channel according to the change of intracellular calcium concentration [12]. Therefore, we hypothesized that the high-calcium microenvironment may cause changes in the expression of related proteins in cells through these calcium receptors, resulting in the transformation of cell phenotype and the formation of the Randall calcium spots, which initiated the pathological process of calculi formation. In order to verify this idea, we compared the expression levels of calcium ion receptor-related proteins STIM1 and Orai1 in renal papillary tissues of patients with calculi and those of noncalculus patients through the GEO gene bank. The results showed that the expression of STIM1 protein in patients with calculi was significantly lower than that in patients without calculi.

## 2. Materials and Methods

### 2.1. Comparison of the Expression Levels of STIM1 and Orai1 in Renal Papillary Tissues between Calculi Patients and Noncalculi Patients

The Randall calcium plaque chip of human renal papillary tissue was found by Gene Expression Omnibus (GEO), and the data number was GSE73680 [13]. GEO2R online analysis system was used to analyze the difference of STIM1 protein and Orai1 protein expression level in renal papilla tissue between calculi patients and noncalculi patients in GSE73680 data set.

### 2.2. Cell Culture

The experimental renal tubular epithelial cell NRK-52E was purchased from Shanghai Cell Bank, Chinese Academy of Sciences. NRK-52E was cultured in an incubator with 5% carbon dioxide at 37°C. They were cultured in the Dulbecco's Modified Eagle's Medium (Hyclone, UT) containing 10% serum (Gibco, Grand Island, NY). The culture medium was changed once every 2-3 days, and the passage was carried out once every 1 week.

### 2.3. Preparation of High-Calcium Medium

To simulate the high-calcium microenvironment in renal papilla of patients with calculus, we prepared high-calcium medium with different concentration gradients to treat NRK-52E cells (including 0.1 mg/mL, 0.3 mg/mL, 0.5 mg/mL, 0.7 mg/mL, and 1.0 mg/mL). A certain amount of anhydrous calcium chloride was dissolved in ultrapure water to prepare a solution with calcium ion concentration of 10 mg/mL. Then, a filter with pore size of 0.22 *μ*m was used to remove potentially pure microorganisms. Different volumes of calcium ion solution were added into 50 mL medium to prepare the high-calcium medium with the above concentration gradient.

### 2.4. Determination of Cell Activity under Different Concentrations of High-Calcium Microenvironment

The well-cultured NRK-52E cells were seeded into a 96-well plate (about 3000 cells per well) and incubated overnight. The NRK-52E cells were treated with different concentrations of high-calcium medium for 24 hours and 48 hours, and each concentration was set with three replicate wells. After high-calcium treatment, 100 *μ*L medium containing 10% CCK-8 was replaced and incubated for 2 hours. Finally, the absorbance of each well at 450 nm was measured with a microplate reader. The untreated group was used as a control, and the percentage of cell viability after treatment with different concentrations of high calcium was calculated.

### 2.5. Determination of Apoptosis

According to the results of cell viability determination, the high-calcium microenvironment of 0.7 mg/mL and 1.0 mg/mL could cause significant changes in cell viability. Therefore, we determined the apoptosis of cells in the high-calcium microenvironment of 0.7 mg/mL and 1.0 mg/mL. The well-cultured NRK-52E cells were seeded into a 6-well plate (about 1 × 10^6^ cells per well) and incubated overnight. The NRK-52E cells in the six-well plate were treated with 0.7 mg/mL and 1.0 mg/mL high-calcium medium for 24 hours and 48 hours, and each concentration was set with three replicate wells. After the high-calcium treatment, the cells were digested with 2.5% trypsin and washed twice with PBS. The cells were resuspended in 200 *μ*L buffer, and 5 *μ*L fluorescein isothiocyanate-Annexin V and 5 *μ*L propidium iodide were added. The cells were incubated at room temperature in dark for 20 minutes. Cell staining was analyzed by flow cytometry. The optimum concentration of high calcium was 0.7 mg/mL.

### 2.6. Detection of the Expression of Cell Phenotype Marker Proteins E-cadherin and OPN and Calcium Channel Proteins STIMl and Orai1

The NRK-52E cells treated with high calcium or shRNA transfected were lysed by RIPA (radioimmunoassay) cell lysate. The protein was separated and extracted by low-temperature centrifuge (4°C, 12000 rpm, centrifugation for 5 minutes), and the supernatant after centrifugation was the extracted total protein. The protein concentration in supernatant was determined by BCA protein concentration determination kit (Beyotime Institute of Biotechnology, China). The proteins with different molecular weights were separated by gel electrophoresis, and then, the protein bands were transferred to polyvinylidene fluoride membranes by membrane transfer solution, and the protein bands were incubated with primary antibody at 4°C overnight: mouse monoclonal *β*-actin (Proteintech, China, 1 : 500), rabbit polyclonal anti-E-cadherin antibody (Boster, China, 1 : 1000), mouse polyclonal anti-OPN antibody (Boster, China, 1 : 1000), rabbit polyclonal anti-STIMl antibody (Boster, China, 1 : 1000), and mouse monoclonal anti-Orai1 antibody (Invitrogen, China, 1 : 1000). Then, the secondary antibody was incubated at room temperature for 1-2 hours and then visualized in chemiluminescence imaging system (Gene Company Limited, China) using enhanced chemiluminescence analysis kit.

### 2.7. Alizarin Red Staining

The well-cultured NRK-52E cells were seeded into a 6-well plate. After the cell density reached 70%-80%, the cells were treated with high calcium for 24 hours and 48 hours and then washed with PBS for 3 times and fixed with 95% ethanol. The fixed cells were stained with alizarin red for 3-5 minutes at room temperature. Then, the excess dye was removed, the staining of calcium salt deposition was observed under the microscope, and the area of staining area was measured by ImageJ software.

### 2.8. Plasmid Transfection

Plasmid-STIM1 and plasmid-shRNA-STIM1 (5′-GATCCC-AGGCTCTCAATGCCACGTCTT-CTCGAG-AAGACGTGGCATTGAGAGCCT-TTTTTGGAT) were synthesized by GENECHEM (Shanghai, China). The well-cultured NRK-52E cells were seeded into a 6-well plate. After the cell density reached 70%-80%, the plasmid was transfected into the cells with Lipofectamine 3000 reagent. Two days after transfection, the transfection efficiency was tested by western blot (WB). The transfected cells were used for subsequent experiments.

### 2.9. Immunofluorescence

The NRK-52E cells treated with high calcium or transfected were washed three times with PBS at 4°C. The washed cells were fixed in 4% paraformaldehyde for 15 minutes, then permeabilized in PBS containing 0.1% Triton X-100 for 30 minutes, and washed again with ice PBS for 3 times. Subsequently, the cells were blocked in 5% bovine serum albumin for 2 hours. Then, the cells were incubated with a mixture of 1% anti-E-cadherin primary antibody and 1% anti-OPN primary antibody overnight at 4°C. The mixture of 0.5% anti-rabbit-FITC and 0.5% anti-mouse-Tex-Red was incubated for 1 hour at room temperature. Then, the nuclei were stained with DAPI. The expression of E-cadherin and OPN was observed under fluorescence microscope.

### 2.10. Determination of Intracellular Calcium Concentration

In this study, we detected the intracellular calcium concentration of NRK-52E cells in different treatment groups by using Best Bio's intracellular calcium detection kit. The F3 staining solution of the above kit was diluted with HBSS buffer at the ratio of 1 : 400. The NRK-52E cells were digested and centrifuged to prepare cell suspension and then washed with HBSS buffer for three times. Finally, the NRK-52E cells were incubated at 37°C for 20 minutes. The cells were washed 2-3 times with HBSS and then resuspended. The distribution of intracellular fluorescence intensity was detected by flow cytometry.

## 3. Results

### 3.1. GEO Database Analysis Showed that the Calcium Channel Protein STIM1 Was Differentially Expressed in Renal Papillary Tissues of Calculi Patients and Noncalculi Patients

As shown in Figures 1(a) and 1(b), the expressions of STIM1 and Orai1 in renal papillary tissues of calculi patients and noncalculi patients were analyzed according to GEO database. According to the statistical analysis of the two protein expression values, the expression of STIM1 protein in calculi patients was significantly lower than that in noncalculi patients, and there was no significant difference in Orai1 protein between calculi patients and noncalculi patients (Figure 1(c)). Therefore, we would explore the role of calcium channel protein STIM1 in the phenotypic transition of renal tubular epithelial cells and calculi formation in this study.

### 3.2. High Concentration of Calcium Inhibited the Activity of NRK-52E Cells and Induced Apoptosis

The effects of different concentrations of high-calcium medium on the activity of NRK-52E cells were explored by CCK-8 experiment. The results are shown in Figure 1(a). In the case of culture for 48 hours, the cell activity of NRK-52E was significantly inhibited when the high-calcium concentration reached 0.7 mg/mL; in the case of culture for 24 hours, the cell activity of NRK-52E was significantly inhibited when the high-calcium concentration reached 1.0 mg/mL. At the same time, the apoptosis rate of NRK-52E cells also increased significantly (Figures 2(b) and 2(c)). Based on the above findings, we simulated the pathological microenvironment of urolithiasis with a high-calcium concentration of 0.7 mg/mL in our follow-up experiments.

### 3.3. Phenotypic Transformation of NRK-52E Cells Occurred after High-Calcium Microenvironment Treatment, and the Expression of Calcium Channel Protein STIM1 Decreased during Phenotypic Transformation

The expression of epithelial marker E-cadherin and osteogenic marker OPN of NRK-52E cells decreased significantly after cultured in 0.7 mg/mL high-calcium medium. The expression of calcium channel proteins STIM1 and Orai1 decreased significantly, especially the difference of STIM1 protein expression (Figures 3(a) and 3(b)). With the increase of high-calcium treatment time, the expression difference of phenotypic marker molecules and calcium channel proteins became more significant. The above results were further verified by RT-PCR analysis (Figure 3(c)).

### 3.4. The Adhesion and Deposition of Calcium Salt on NRK-52E Cells after Phenotypic Transformation Increased Significantly

We identified the adhesion and deposition of calcium salts by NRK-52E cells by alizarin red staining. As shown in Figures 3(d) and 3(e), the NRK-52E cells after high-calcium treatment had significantly more alizarin red staining areas, and the alizarin red staining areas increased with the increase of culture time.

### 3.5. Downregulating the Expression of STIM1 Protein Promoted the Phenotypic Transformation of the NRK-52E Cells

We transfected NRK-52E cells with shRNA plasmid to silence the expression of STIM1 protein. Western blot analysis showed that the expression of E-cadherin was significantly decreased and the expression of OPN was significantly increased in NRK-52E cells after silencing STIM1 protein, which was similar to NRK-52E cells treated with high-calcium microenvironment, and both of them had phenotypic transformation (Figures 4(a) and 4(b)). Immunofluorescence analysis further confirmed that silencing the protein expression of STIM1 could promote the phenotypic transformation of NRK-52E cells (Figure 4(c)).

### 3.6. Upregulating the Expression of STIM1 Protein Promoted the Increase of the Expression of the Epithelial Phenotype Marker E-cadherin of the NRK-52E Cells

The expression of STIM1 protein in the NRK-52E cells was promoted by plasmid transfection. We found that the expression of E-cadherin was significantly increased in the NRK-52E cells after overexpression of STIM1 protein, but the expression of OPN was not significantly changed (Figures 5(a) and 5(b)). Immunofluorescence assay showed the same results (Figure 5(c)).

### 3.7. Downregulating the Expression of STIM1 Protein and the High-Calcium Microenvironment Both Caused a Significant Decrease in Calcium Ion Content in the NRK-52E Cells

As shown in Figures 5(d) and 5(e), the calcium ion content of NRK-52E cells in different treatment groups was shown. Compared with the control group, the intracellular calcium concentration of the NRK-52E cells in the downregulated group decreased significantly. The intracellular calcium concentration of most NRK-52E cells in the high-calcium treatment group decreased significantly. The calcium concentration in the NRK-52E cells in the upregulation group was slightly increased, but there was no significant difference compared with the control group.

## 4. Discussion

The causes of urinary calculi are quite complex, and Randall's plaque (RP) theory is one of the theories widely recognized by relevant scholars [8, 14, 15]. RP is a calcium salt deposit originated from renal papillary interstitium, which is considered as a key role site for calculi formation and anchoring [16]. The main component of RP is hydroxyapatite (the main component of bone). Researchers believe that the process of calculi formation may be related to the process of osteogenesis [17]. The previous research of our group found that the expression of osteogenic marker OPN in renal tubular epithelial cells increased significantly, while the epithelial marker E-cadherin decreased significantly [18]. Therefore, we believed that the renal tubular epithelial cells were undergoing phenotypic transformation: from epithelial cells to osteoblasts. We further found that the phenotype-transformed epithelial cells had significant calcium attachment ability, and thus, we considered that it was the cause of RP [19].

Pathological examination of renal papilla indicates that high calcium, hypoxia, and inflammation were important components of the lithogenic microenvironment and might be the important inducement to induce the formation of RP, among which high-calcium microenvironment is the most common in pathological specimens of patients with calculi [20]. STIM1 is a single transmembrane protein located in the endoplasmic reticulum, a sensor of calcium ion concentration in the endoplasmic reticulum, and a regulatory protein for the opening of calcium ion channels on the cell membrane surface [21]. STIM1 can regulate the activation of multiple pathways by sensing changes in the concentration of calcium ions in the endoplasmic reticulum [11, 22]. Therefore, we speculate that the high-calcium microenvironment may induce the formation of RP through STIM1 protein [23]. Interestingly, the analysis from the public database reveals that the expression status of STIM1 was significantly higher in control normal tissue than stone plaque tissue, and this result aroused our interests.

In this study, we verified the phenotypic transformation of the NRK-52E cells in high-calcium microenvironment through the expression changes of phenotypic markers. As shown in the above results, the expression of epithelial phenotype marker E-cadherin in NRK-52E cells decreased significantly after high-calcium treatment, while the expression of osteogenic marker OPN increased significantly. At the same time, we found that the expression of STIM1 protein also decreased significantly during phenotypic transformation. In order to explore whether there is a causal relationship between the low expression of STIM1 protein and the phenotype transformation of NRK-52E cells, we upregulated/downregulated the expression of STIM1 protein in the NRK-52E cells by plasmid transfection and found that the phenotype transformation of the NRK-52E cells also occurred when the expression of STIM1 protein was downregulated. These results fully proved that the high-calcium microenvironment can induce phenotypic transformation of the NRK-52E cells by regulating the expression of STIM1 protein. In addition, we also further measured the intracellular calcium ion concentration of the NRK-52E cells in a high-calcium microenvironment, and the results showed that the intracellular calcium concentration of some NRK-52E cells decreased, which was similar to that of the NRK-52E cells with downregulation of STIM1 protein expression.

There are still some limitations in this study: Firstly, our study only revealed the role of STIM1 protein in phenotypic transformation, but the mechanism by which STIM1 protein plays a role needs further research to explore. Secondly, our study only involved the phenotypic transformation stage of the NRK-52E cells and lacked the verification of the subsequent kidney calculi formation process, which need to be verified by subsequent animal experiments in vivo. Finally, due to the current reports on STIM1 protein mostly focus on its role as a calcium channel regulatory protein, there are no reports showing the relationship between STIM1 protein expression and kidney calculi formation or phenotypic transformation. Hence, more studies are needed to verify our results.

## 5. Conclusion

STIM1 protein plays an important role in promoting the phenotypic transformation of NRK-52E cells in the high-calcium microenvironment and may be an important pathway protein in the formation of calcium-containing kidney calculi.

## Figures and Tables

**Figure 1:** (a) The expressions of STIM1 in renal papillary tissues of calculi patients and noncalculi patients were analyzed according to GEO database. (b) The expressions of Orai1 in renal papillary tissues of calculi patients and noncalculi patients were analyzed according to GEO database. (c) The expression of STIM1 protein in calculi patients was significantly lower than that in noncalculi patients; there was no significant difference in Orai1 protein between calculi patients and noncalculi patients.

**Figure 2:** (a) The NRK-52E cells were treated with the different concentrations of high-calcium medium, and then, the activity of the NRK-52E cells was explored by CCK-8 experiment. (b and c) The apoptosis rate of the NRK-52E cells was determined by flow cytometry when treated with high-calcium medium.

**Figure 3:** (a and b) The NRK-52E cells were treated with the concentrations of high-calcium medium (0.7 mg/mL), and then, the expression of calcium channel protein (STIM1 and Orai1) and phenotypic marker proteins (E-cadherin and OPN) were determined by western blot. (c) The above results were further verified by RT-PCR analysis. (d and e) The adhesion and deposition of calcium salt on NRK-52E cells increased significantly, when the NRK-52E cells were treated with the concentrations of high-calcium medium (0.7 mg/mL).

**Figure 4:** (a and b) Western blot analysis showed that the expression of E-cadherin was significantly decreased and the expression of OPN was significantly increased in the NRK-52E cells after silencing STIM1 protein, which was similar to the NRK-52E cells treated with high-calcium microenvironment. (c) Immunofluorescence analysis further confirmed the above results.

**Figure 5:** (a and b) Western blot analysis showed that the expression of E-cadherin was significantly increased in the NRK-52E cells after overexpression of STIM1 protein. (c) Immunofluorescence assay showed the same results. (d and e) The calcium ion content of the NRK-52E cells in different treatment groups was shown.

## Data Availability

Source data support of this study is available from the corresponding author by email upon reasonable request.

## References

[1] Rule A. D., Lieske J. C., Pais V. M. (2020). Management of kidney stones in 2020. *JAMA*.

[2] Ferraro P. M., Bargagli M., Trinchieri A., Gambaro G. (2020). Risk of kidney stones: influence of dietary factors, dietary patterns, and vegetarian–vegan diets. *Nutrients*.

[3] Zeng G., Mai Z., Xia S. (2017). Prevalence of kidney stones in China: an ultrasonography based cross-sectional study. *BJU International*.

[4] Tahbaz R., Schmid M., Merseburger A. S. (2018). Prevention of kidney cancer incidence and recurrence. *Current Opinion in Urology*.

[5] Goka S. Q., Copelovitch L. (2020). Prevention of recurrent urinary stone disease. *Current opinion in pediatrics*.

[6] Caudarella R., Tonello L., Rizzoli E., Vescini F. (2011). Predicting five-year recurrence rates of kidney stones: an artificial neural network model. *In: Archivio Italiano di Urologia e Andrologia*.

[7] Okada A., Hamamoto S., Taguchi K. (2018). Kidney stone formers have more renal parenchymal crystals than non-stone formers, particularly in the papilla region. *BMC Urology*.

[8] Evan A. P., Lingeman J. E., Coe F. L. (2003). Randall’s plaque of patients with nephrolithiasis begins in basement membranes of thin loops of Henle. *Journal of Clinical Investigation*.

[9] Winfree S., Weiler C., Bledsoe S. B. (2021). Multimodal imaging reveals a unique autofluorescence signature of Randall’s plaque. *Urolithiasis*.

[10] Xiaoyan Y. U., BAO J., CUI X. (2020). Pyrrolidinedithiocarbamic acid ammonium salt inhibits apoptosis and phenotypic transformation of co-culture of myeloma cells and renal tubular epithelial cells by reducing the secretion of light chain protein. *Iranian Journal of Public Health*.

[11] Roos J., DiGregorio P. J., Yeromin A. V. (2005). STIM1, an essential and conserved component of store-operated Ca 2+ channel function. *Journal of Cell Biology*.

[12] Nguyen N. T., Ma G., Lin E. (2018). CRAC channel-based optogenetics. *Cell Calcium*.

[13] Edgar R., Domrachev M., Lash A. E. (2002). Gene Expression Omnibus: NCBI gene expression and hybridization array data repository. *Nucleic Acids Research*.

[14] Khan S. R., Canales B. K., Dominguez-Gutierrez P. R. (2021). Randall’s plaque and calcium oxalate stone formation: role for immunity and inflammation. *Nature Reviews Nephrology*.

[15] Stoller M. L., Low R. K., Shami G. S., McCormick V. D., Kerschmann R. L. (1996). High resolution radiography of cadaveric Kidneys. *Journal of Urology*.

[16] Evan A. P., Coe F. L., Lingeman J. E. (2007). Mechanism of formation of human calcium oxalate renal stones on Randall’s plaque. *The Anatomical Record: Advances in Integrative Anatomy and Evolutionary Biology*.

[17] Bhuskute N. M., Yap W. W., Wah T. M. (2009). A retrospective evaluation of Randall’s plaque theory of nephrolithiasis with CT attenuation values. *European Journal of Radiology*.

[18] HE D. E. N. G., WANG S. H. A. O. G. A. N. G., JIA Z. H. A. O. H. U. I. (2015). Calcium ions promote primary renal epithelial cell differentiation into cells with bone-associated phenotypes via transforming growth factor-*β*1-induced epithelial-mesenchymal transition in idiopathic hypercalciuria patients. *Molecular Medicine Reports*.

[19] He D., Lu Y., Hu H. (2015). The wnt11 signaling pathway in potential cellular EMT and osteochondral differentiation progression in nephrolithiasis formation. *International Journal of Molecular Sciences*.

[20] Li L., Peng Y., Liu M. (2019). Apoptosis of human kidney epithelial cells induced by high oxalate and calcium oxalate monohydrate is apurinic/apyrimidinic endonuclease 1 pathway dependent and contributes to kidney stone formation. *Discovery Medicine*.

[21] Clapham D. E. (2009). A STIMulus package puts orai calcium channels to work. *Cell*.

[22] Zheng H., Zhou M. H., Hu C. (2013). Differential roles of the C and N termini of Orai1 protein in interacting with stromal interaction molecule 1 (STIM1) for Ca2+ release-activated Ca2+ (CRAC) channel activation. *Journal of Biological Chemistry*.

[23] Tsvilovskyy V., Solís-López A., Schumacher D. (2018). Deletion of Orai2 augments endogenous CRAC currents and degranulation in mast cells leading to enhanced anaphylaxis. *Cell Calcium*.

